# Study on the Effect and Mechanism of Antibacterial Adhesive Hydrogel on Wound Healing

**DOI:** 10.1155/2021/8212518

**Published:** 2021-11-30

**Authors:** Xiaodong Wang, Xuehong Pan, Nana Zhao, Defang Chen

**Affiliations:** ^1^Department of Medical Cosmetology, Yidu Central Hospital of Weifang, Weifang, Shandong Province, China; ^2^Department of Cardiothoracic Surgery, Yidu Central Hospital of Weifang, Weifang, Shandong Province, China; ^3^Outpatient Department, Jinan Central Hospital, Jinan, Shandong Province, China

## Abstract

Bleeding and infection can cause significant increases in mortalities. Hydrogel sealants have attracted extensive attention for their ability to control bleeding. In this study, the adjuvant treatment with antibacterial adhesive hydrogel dressings was applied to patients with deep second-degree burns/scalds. The traditional medical dressing was regarded as control adjuvant treatment. The results indicated that the total positive rate of bacteria in wound secretions and the pain during dressing change in patients who used antibacterial adhesive hydrogel dressings were significantly reduced. The number of fibroblasts and new capillaries in the granulation tissue of the wound increased, and the patient's wound healing is accelerated. The overall clinical effectiveness has been significantly improved. It is proven that the antibacterial adhesive hydrogel dressing has a significant effect on wound healing.

## 1. Introduction

The skin is the human body's largest natural barrier, which keeps the internal environment stable and protects tissues and organs from chemical substances and physical and pathogenic microorganisms [1]. Skin damage caused by abrasion after falling and clinical incision after surgery are the most common wounds in real life [2]. In clinic, most wounds are sterilized with 75% alcohol or iodine, followed by covering with cotton gauzes [1–3]. Fixed cotton gauze dressing needs to be taped, and sometimes the skin is allergic to the tape material. Compared with the wounds at flat areas of the human body, it is still challenging to treat the wounds at special areas such as joints, popliteal fossae, axillae, and muscle folds. Therefore, wound treatment is still challenging in special areas because of inevitable movements and difficult fixation [3–6]. To this end, designing a stretchable, adhesive, antibacterial, and biocompatible dressing is of great clinical significance.

Hydrogels have been considered good candidates for wound dressing because of their good flexibility and biocompatibility. In recent years, adhesive hydrogels with good biocompatibility, flexibility, and wettability have been widely used in wound dressings, tissue adhesion, biosensing, and other fields [7]. Hydrogel is a flexible material composed of a hydrophilic polymer network, which can swell in water but not easy to dissolve [8]. Therefore, the hydrogel can absorb a lot of water [9], provide a humid environment for callus cells, accelerate collagen synthesis, and promote wound healing. In addition, the hydrogel has a good elastic structure [10], and it can reduce irritation to wounds and inflammation in adjacent areas. Nevertheless, colloidal dressings that have no antibacterial effect are susceptible to bacterial erosion and deterioration [11]. As we all know, pathogenic bacterial infection is the main reason contributing to the impediment of wound healing. To address this issue, many studies have set to explore adhesive hydrogels with antibacterial effects on animals [12]. Studies have indicated that the introduction of inorganic nanometal particles, organic antibacterial agents, chitosan, and other materials into the hydrogel can enhance the antibacterial adhesion performance and bactericidal performance [13]. However, the effect and mechanism of this antibacterial adhesive hydrogel on wound healing in clinical patients are still in the early stage of exploration. At present, most of the wounds of hospitalized patients due to burns and scalds are II degree deep [14]. It also often causes bacterial infections due to incorrect handling, leading to poor treatment effect. Herein, this study mainly concentrated on patients with deep second-degree burns/scalds as experimental subjects and attempted to explore the effect and specific mechanism of antibacterial adhesive hydrogel on promoting wound healing in patients, to provide a reference for clinical treatment of deep second-degree burns/scalds.

## 2. Materials and Methods

### 2.1. Research Objects

Patients with deep second-degree burns/scalds admitted to our hospital for treatment from June 2019 to May 2020 were selected. Inclusion criteria were as follows: (1) skin burns/scalds caused by II degree hydrothermal fluid (water) or flame (including shallow II degree, deep II degree, and mixed II degree); (2) burn/scald total body surface area (TBSA) ≤ 30% of mild to moderate degree, no symptoms of infection on the wound, and nonjoint parts; and (3) complete clinical data, aged 20 to 59 years old, and voluntarily joining the study. Exclusion criteria were as follows: (1) contraindications of analgesic and sedative drugs, (2) women during lactation or pregnancy, (3) accompanied by clearly infectious wounds, (4) long-term use of hormones before injury, (5) combined diabetes and mental illness, (6) patients with liver and kidney dysfunction, (7) those with severe mental illness, and (8) those who cannot communicate in language. A total of 88 patients were eligible for inclusion and exclusion. They were divided into the observation group (*n* = 44) and control group (*n* = 44) at random. The ratio of men to women in the observation group was 26 : 18. The age ranges from 14 to 72 years old, with an average age of 44.64 ± 14.35 years. The ratio of male to female in the control group is 25 : 19. The age ranged from 15 to 71 years, with an average of 46.18 ± 14.13 years. Age, gender, and wound condition were compared between the two groups (see Figures 1 and 2), and good balance (*P* > 0.05) was also comparable. This study has been approved by the medical ethics committee of our hospital. All patients signed an informed consent form.

### 2.2. Methods

After admission, all patients were cleaned and disinfected with 1% iodophor solution, blood clots were removed, and blisters were removed. Then, rinse the wound with sterile normal saline. Let the wound dry with a sterile cotton ball. After routine debridement, 1% sulfadiazine silver cold cream (produced by Tianjin Jinyao Pharmaceutical Co., Ltd.) was applied and spread evenly on the wound surface. The smearing area should be slightly larger than the area covering the wound. The coating thickness is about 1.5-2 mm. Then, the control group was wrapped with petrolatum medical gauze. Dressing is changed once a day. The observation group used antibacterial adhesive hydrogel dressings, and the dressing contains inorganic nanometal particles, organic antibacterial agents, chitosan, and other materials, prepared by China Bristol-Myers Squibb Medical Co., Ltd. Cover and bandage the wound with hydrogel dressing, and change the dressing on the wound every other day.

### 2.3. Observation Indicators

#### 2.3.1. The Total Positive Rate of Bacteria in Wound Secretions

Before treatment and 6 days after treatment, samples of wound secretions were collected by the smearing method and sent to the bacteria room for culture. Use Takara's bacterial DNA kit to extract bacterial DNA template solution, and perform nano-PCR amplification. The reaction system is 12 *μ*L, with details as follows: 2~NanoPCRBufer 6 *μ*L, 25 mmol/L MgC1_2_ 1 L, 0.5 *μ*L each of the upstream and downstream primers of 50 *μ*mol/L, 5 U/*μ*L Taq enzyme 0.2 gL, ddH_2_O 3.2 *μ*L, and 1 *μ*L of DNA template. The amplification conditions were 95°C for 5 min, 95°C for 25 s, 53°C for 45 s, 70°C for 40 s, and 30 cycles of 72°C for 10 min. Test specimens for bacteria such as Acinetobacter baumannii, Proteus proteus, Escherichia coli, Pseudomonas aeruginosa, and Staphylococcus epidermidis. Calculate the positive detection rate of bacteria.

#### 2.3.2. The Number of New Capillaries and Fibroblasts in the Granulation Tissue

3 d and 6 d after treatment, observe the tissue condition of the patient after wound repair under a light microscope. And randomly select 5 high-power lens fields, count the number of fibroblasts and new capillaries, and calculate its mean.

#### 2.3.3. Pain and Wound Healing Time

The visual analogue scale (VAS) was used to evaluate the pain before treatment and during medication. The score is 0-10 points. The higher the score, the stronger the pain. From the day of treatment until the wound is completely healed, that is counted as wound healing time.

#### 2.3.4. Clinical Efficacy

The clinical efficacy of the patients was evaluated after 2 weeks of treatment: invalid: there is no change in the wound, or the wound area is smaller than 25% before treatment, with more secretions; effective: the wound area is reduced by 25%~50%, with significant reduction in secretions; significantly effective:wound reduction > 50%, and there is almost no secretion; and cure: the wound is completely epithelialized, the color is reddish, dryness is observed, there is no exudation, the surface becomes smooth, and no scabs exist. The total effective rate of wound healing = (effective + markedly effective + healing)/total number of cases × 100%.

### 2.4. Statistical Analysis

SPSS 19.0 software was utilized for data analysis. Counting data is expressed as frequency. The chi-square (*χ*^2^) test is performed disorderly. Perform the rank sum (*Z*) test in an orderly manner. The measurement data is expressed as the mean ± standard deviation (mean ± SD). The *t*-test was used to compare the two groups. The difference was statistically significant with *P* < 0.05.

## 3. Results and Discussion

### 3.1. Comparison of the Positive Rate of Bacteria in Wound Secretions between the Two Groups

Before therapy, bacterial culture results of wound secretions in both groups were negative. Six days after treatment, the positive detection rate of bacteria in wound secretions of the observation group was lower than that of the control group. The difference is statistically significant (*P* < 0.05). See Table 1 and Figure 3.

### 3.2. The Number of Fibroblasts and the Number of New Capillaries in the Granulation Tissue of the Wound on the 3rd and 6th Day of Treatment in the Two Groups

The number of fibroblasts and new capillaries in the wound granulation tissue of the observation group was significantly higher than that of the control group on the 3rd and 6th day of treatment. The difference is statistically significant (*P* < 0.05). See Table 2 and Figure 4.

### 3.3. Comparison of Pain Scores and Wound Healing Time between the Two Groups

In terms of the pain score, VAS scores were compared between the two groups before treatment (*P* < 0.05); however, the VAS score of the observation group when applying medicine on the wound was lower than that of the control group (*P* < 0.05). In terms of healing time, the observation group is faster than the control group (*P* < 0.05). See Table 3 and Figures 5 and 6.

### 3.4. Comparison of Clinical Efficacy between the Two Groups

The clinical efficacy rate of the observation group (93.18%) was higher than that of the control group (81.18%). The difference is statistically significant (*P* < 0.05). See Table 4 and Figure 7. The typical wound healing process of the observation group is shown in Figure 8.

### 3.5. Discussion

The pathological characteristics of burns and scalds are mainly the damaged cortex [15]. In particular, bleeding-induced infection is one of the significant causes of complications in tissue regeneration, resulting in inflammatory response and delayed healing in wounds [4, 5]. Hydrogel-based hemostatic materials have drawn significant attention in recent years because they act as sealants to control bleeding [1, 3, 6, 7], which provides a barrier against infection by microorganisms [4, 8, 9] and creates a suitable microenvironment for accelerated wound healing. At present, there are many kinds of external wound dressings. A good topical dressing should not only prevent wound infection but also provide an optimal healing environment for wound healing. Meanwhile, it should have the characteristics of convenient use, safety, fast absorption, and low side effects [15]. The existing conventional medical dressings have poor water absorption, poor congeniality, and strong adhesion to wounds. When applied to wounds that damage the dermis, often due to excessive wound exudate, they can cause the dressing to adhere to wound secretions [3]. Thus, choosing the right wound dressing is extremely important.

Good topical antibacterial drugs are very important for wound healing. 1% sulfadiazine silver cold cream is the most widely used external medicine for burns/scalds. It has been used clinically for more than 40 years, but due to the emergence of bacterial resistance, its bactericidal ability is significantly reduced [16]. Currently, hydrogel sealants have attracted extensive attention for their ability to control bleeding. It has the same physical properties as human living tissues, such as adhesion, elasticity, and low interfacial tension [17, 18], and also, it can reduce irritation to surrounding tissues [19], reduce negative immune response, and increase the residence time of the drug and the permeability of the tissue [20]. In this study, an antibacterial adhesive hydrogel dressing was used to treat the wounds of burn/scald patients and compared with the adjuvant treatment of traditional medical dressings for wound healing. The results showed that the total positive rate of bacteria in wound secretions and the pain during dressing change were significantly reduced. In addition, the number of fibroblasts and new capillaries in the granulation tissue of the patient's wound increased significantly, and the overall clinical effectiveness has been significantly improved. This shows that the antibacterial adhesive hydrogel dressing has a significant auxiliary effect on wound healing. Its mechanism is analyzed. The antibacterial adhesive hydrogel dressing used herein is made of inorganic nanometal particles, with ze as a carrier, having the sustained release effect of drugs. Nano-ultrafine particles are made by nanotechnology using sterile medical gauze, which can be oxidized to silver ions (Ag+), and Ag+ can promote the interaction of the sulfhydryl group of the protein on the bacterial cell membrane to attach, inhibit DNA replication, and then realize the antibacterial effect [21]. With chitosan under weakly acidic conditions, some of the amino groups on chitosan will be protonated and converted into quaternary ammonium salt and inhibit the growth of microorganisms [22], exerting a significant antibacterial effect on promoting wound healing. Previous evidences have shown that a composite hydrogel containing chitosan, showing positive antibacterial activity against Escherichia coli, can promote the proliferation of fibroblasts [23], which is conducive to wound healing. In addition, chitosan also has the ability to coordinate and bind metal and can enhance the antibacterial effect of inorganic nanometal particles and reduce the toxicity of inorganic nanometal particles [24]. Recent studies have confirmed that hydrogel dressings containing organic antibacterial agents can effectively reduce bacterial infections, be conducive to the growth of granulation, and stimulate the wound to heal faster [25]. Hydrogel dressings can provide a suitable environment for cell growth, help promote the growth of new capillaries, and speed up wound healing. When the hydrogen bonds between the water molecules in the hydrogel and the adhesion groups of the above-mentioned materials interact, it can greatly weaken the adhesion of the dressing to the skin, thereby reducing the pain or secondary injury caused by the adhesion of the dressing and the secretion when the patient changes dressing. Nonetheless, allergenicity and cytotoxicity could not be underestimated in the practical performances. Therefore, more efforts are still anticipated to develop new or advanced antibacterial adhesive gels.

## 4. Conclusion

This study is the first to explore the clinical effect of antibacterial adhesive hydrogel dressings on wound healing. The results show that nanoparticle-containing antibacterial adhesive hydrogel dressings can reduce the positive rate of wound bacteria and also promote the growth of fibroblasts and new blood vessels in the wound tissue, effectively alleviating the pain caused to patients when changing dressings. Our findings collectively provide a new reference basis for clinical treatment of wounds.

## Figures and Tables

**Figure 1:** Comparison of wound types between the two groups.

**Figure 2:** Comparison of average TBSA between the two groups.

**Figure 3:** The positive rate of bacteria in the two groups.

**Figure 4:** The number of fibroblasts and the number of new capillaries in the granulation tissue of the two groups on the 3rd and 6th day of treatment. Compared with the control group (^a^*P* < 0.05) on the 3rd day of treatment and (^b^*P* < 0.05) on the 6th day of treatment.

**Figure 5:** Compared with the treatment of the control group (^∗^*P* > 0.05) and compared with the control group when changing the dressing (^#^*P* < 0.05).

**Figure 6:** Comparison of wound healing time with the control group (^∗^*P* < 0.05).

**Figure 7:** Comparison of clinical efficacy between the observation group (*n* = 44) and control group (*n* = 44) (*P* < 0.05).

**Figure 8:** The treatment process of the wound surface after the scald of the patient: (a) before the treatment of the scalded patient with the antibacterial adhesive hydrogel; (b) the 3rd day after the treatment with the antibacterial adhesive hydrogel; (c) after the treatment with the antibacterial adhesive hydrogel (6 d); (d) 12 days after treatment with the antibacterial adhesive hydrogel.

**Table 1:** The positive rate of bacteria in wound secretions after 6 days of treatment in the two groups (*n*, %).

Group	*n*	Acinetobacter baumannii	Staphylococcus aureus	Escherichia coli	Pseudomonas aeruginosa	Proteus	Staphylococcus epidermidis
Observation	44	0 (0.00)	1 (2.27)	0 (0.00)	1 (2.27)	0 (0.00)	1 (2.27)
Control	44	2 (4.55)	3 (6.82)	1 (2.27)	4 (9.09)	2 (4.55)	3 (6.82)
*χ* ^2^					13.019		
*P*					0.043		

**Table 2:** The number of fibroblasts and the number of new capillaries in the granulation tissue of the wound on the 3rd and 6th day of treatment (mean ± SD).

Group	*n*	Number of fibroblasts		Number of new capillaries	
		Treatment 3 d	Treatment 6 d	Treatment 3 d	Treatment 6 d
Observation	44	125.32 ± 12.87	165.31 ± 15.68	30.12 ± 5.34	3925 ± 5.16
Control	44	102.69 ± 10.23	134.23 ± 13.22	24.34 ± 4.67	32.27 ± 4.75
*t*		9.131	10.050	5.405	6.602
*P*		<0.001	<0.001	<0.001	<0.001

**Table 3:** Pain scores and wound healing time in the two groups (mean ± SD).

Group	*n*	VAS score (points)		Wound healing time (d)
		Before therapy	When the medicine is applied on the wound	
Observation	44	7.16 ± 1.93	2.38 ± 0.54	17.15 ± 3.18
Control	44	7.09 ± 1.76	4.62 ± 1.25	20.63 ± 4.43
*t*		0.178	10.910	4.233
*P*		0.859	<0.001	<0.001

**Table 4:** Comparison of clinical efficacy between the two groups (*n*, %).

Group	*n*	Cure	Significantly effective	Effective	Invalid
Observation	44	15 (34.09)	18 (40.91)	8 (18.18)	3 (6.82)
Control	44	12 (27.27)	17 (38.64)	7 (15.91)	8 (18.18)
*Z*			-2.686		
*P*			0.007		

## Data Availability

All the raw data not included in the article is available from the corresponding author on reasonable request.

## References

[1] Deng Z. H., Yin J. J., Luo W. (2018). The effect of earthworm extract on promoting skin wound healing. *Bioscience Reports*.

[2] Brohem C. A., da Silva Cardeal L. B., Tiago M., Soengas M. S., de Moraes Barros S. B., Maria-Engler S. S. (2011). Artificial skin in perspective: concepts and applications. *Pigment Cell & Melanoma Research*.

[3] Mason S. A., Nathens A. B., Byrne J. P. (2017). Trends in the epidemiology of major burn injury among hospitalized patients: a population-based analysis. *The Journal of Trauma and Acute Care Surgery*.

[4] Haalboom M. (2018). Chronic wounds: innovations in diagnostics and therapeutics. *Current Medicinal Chemistry*.

[5] Francesko A., Petkova P., Tzanov T. (2018). Hydrogel dressings for advanced wound management. *Current Medicinal Chemistry*.

[6] Moiemen N. S., Shale E., Drysdale K. J., Smith G., Wilson Y. T., Papini R. (2011). Acticoat dressings and major burns: systemic silver absorption. *Burns*.

[7] Zhao X., Guo B., Wu H., Liang Y., Ma P. X. (2018). Injectable antibacterial conductive nanocomposite cryogels with rapid shape recovery for noncompressible hemorrhage and wound healing. *Nature Communications*.

[8] Shi Z., Gao X., Ullah M. W., Li S., Wang Q., Yang G. (2016). Electroconductive natural polymer-based hydrogels. *Biomaterials*.

[9] Ahmed E. M. (2015). Hydrogel: preparation, characterization, and applications: a review. *Journal of Advanced Research*.

[10] Matricardi P., Di Meo C., Coviello T., Hennink W. E., Alhaique F. (2013). Interpenetrating polymer networks polysaccharide hydrogels for drug delivery and tissue engineering. *Advanced Drug Delivery Reviews*.

[11] Rauner N., Meuris M., Zoric M., Tiller J. C. (2017). Enzymatic mineralization generates ultrastiff and tough hydrogels with tunable mechanics. *Nature*.

[12] Nimal T. R., Baranwal G., Bavya M. C., Biswas R., Jayakumar R. (2016). Anti-staphylococcal activity of injectable nano tigecycline/chitosan-PRP composite hydrogel using Drosophila melanogaster model for infectious wounds. *ACS Applied Materials & Interfaces*.

[13] Qu J., Zhao X., Liang Y., Zhang T., Ma P. X., Guo B. (2018). Antibacterial adhesive injectable hydrogels with rapid self-healing, extensibility and compressibility as wound dressing for joints skin wound healing. *Biomaterials*.

[14] Esteban-Vives R., Corcos A., Choi M. S. (2018). Cell-spray auto-grafting technology for deep partial-thickness burns: problems and solutions during clinical implementation. *Burns*.

[15] Green B. (2013). Making an informed decision: how to choose the correct wound dressing. *Professional Nursing Today*.

[16] Boucard N., Viton C., Agay D. (2007). The use of physical hydrogels of chitosan for skin regeneration following third-degree burns. *Biomaterials*.

[17] Ahmadian S., Ghorbani M., Mahmoodzadeh F. (2020). Silver sulfadiazine-loaded electrospun ethyl cellulose/polylactic acid/collagen nanofibrous mats with antibacterial properties for wound healing. *International Journal of Biological Macromolecules*.

[18] Elviri L., Bianchera A., Bergonzi C., Bettini R. (2017). Controlled local drug delivery strategies from chitosan hydrogels for wound healing. *Expert Opinion on Drug Delivery*.

[19] Schreml S., Szeimies R. M., Prantl L., Landthaler M., Babilas P. (2010). Wound healing in the 21st century. *Journal of the American Academy of Dermatology*.

[20] Bhattarai N., Gunn J., Zhang M. (2010). Chitosan-based hydrogels for controlled, localized drug delivery. *Advanced Drug Delivery Reviews*.

[21] Amsden B. (2015). Novel biodegradable polymers for local growth factor delivery. *European Journal of Pharmaceutics and Biopharmaceutics*.

[22] Xu W., Dong S., Han Y., Li S., Liu Y. (2018). Hydrogels as antibacterial biomaterials. *Current Pharmaceutical Design*.

[23] Tsao C. T., Chang C. H., Lin Y. Y. (2010). Antibacterial activity and biocompatibility of a chitosan-*γ*-poly(glutamic acid) polyelectrolyte complex hydrogel. *Carbohydrate Research*.

[24] Archana D., Dutta J., Dutta P. K. (2013). Evaluation of chitosan nano dressing for wound healing: characterization, in vitro and in vivo studies. *International Journal of Biological Macromolecules*.

[25] Li S., Dong S., Xu W. (2018). Antibacterial hydrogels. *Advanced Science*.

[26] Heunis T. D., Smith C., Dicks L. M. (2013). Evaluation of a nisin-eluting nanofiber scaffold to treat Staphylococcus aureus-induced skin infections in mice. *Antimicrobial Agents and Chemotherapy*.

